# Relationships between Personality Traits and Brain Gray Matter Are Different in Risky and Non-risky Drivers

**DOI:** 10.1155/2022/1775777

**Published:** 2022-04-05

**Authors:** Laura Mas-Cuesta, Sabina Baltruschat, Antonio Cándido, Andrés Catena

**Affiliations:** ^1^Mind, Brain and Behavior Research Center, Campus de Cartuja s/n, University of Granada, 18011 Granada, Spain; ^2^Cardiff University Brain Research Imaging Centre, Maindy Rd, Cardiff CF24 4HQ, UK; ^3^School of Psychology, University of Granada, Campus de Cartuja s/n, 18011 Granada., Spain

## Abstract

Personality traits such as impulsivity or sensitivity to rewards and punishments have been associated with risky driving behavior, but it is still unclear how brain anatomy is related to these traits as a function of risky driving. In the present study, we explore the neuroanatomical basis of risky driving behavior and how the level of risk-taking influences the relationship between the traits of impulsivity and sensitivity to rewards and punishments and brain gray matter volume. One hundred forty-four participants with different risk-taking tendencies assessed by real-life driving situations underwent MRI. Personality traits were assessed with self-report measures. We observed that the total gray matter volume varied as a function of risky driving tendencies, with higher risk individuals showing lower gray matter volumes. Similar results were found for volumes of brain areas involved in the reward and cognitive control networks, such as the frontotemporal, parietal, limbic, and cerebellar cortices. We have also shown that sensitivity to reward and punishment and impulsivity are differentially related to gray matter volumes as a function of risky driving tendencies. Highly risky individuals show lower absolute correlations with gray matter volumes than less risk-prone individuals. Taken together, our results show that risky drivers differ in the brain structure of the areas involved in reward processing, cognitive control, and behavioral modulation, which may lead to dysfunctional decision-making and riskier driving behavior.

## 1. Introduction

Risky driving styles, characterized by driving over the speed limit, not paying attention to traffic, driving under the influence of alcohol or drugs, or not wearing a seat belt or helmet, are behaviors associated with a history of traffic offenses [1, 2] and are, in part, responsible for traffic accident fatalities that rank eighth among the causes of mortality worldwide [3, 4]. Certain personality traits, such as impulsivity and sensitivity to rewards and punishments, have been linked to risky driving behavior styles [5, 6]. It seems that the brain systems related to these personality traits show a dysfunctional interaction when making risky decisions [7]. However, there is still a knowledge gap regarding the neuroanatomical bases of risky driving and the relationships between brain anatomy and personality traits such as sensitivity to reward and punishment or preference for immediate versus delayed rewards. Our main aim was to address this gap using a large sample of individuals with different risk tendencies assessed using self-reported real-life driving behaviors.

The brain networks supporting the processing of the subjective value of rewards and punishments and those involved in conflict monitoring in decision-making have been linked to a risky behavior. These networks are located in brain regions such as the striatum, the orbitofrontal cortex (OFC), superior and posterior parietal cortex, the lateral prefrontal cortex (LPFC), the medial temporal lobe, the insula, or the anterior cingulate cortex (ACC) [8–14]. Only a few recent studies have investigated the relationship between risky driving behavior and the volume of brain gray matter of these structures. In a study with people with multiple sclerosis, Dehning et al. [15] found that the size of the third ventricle, an indicator of thalamic atrophy, was significantly correlated with traffic rule violations and predicted a significant portion of the variance in traffic offenses. Kwon et al. [16] observed, in a computerized driving task, that more risky adolescents did not show differences in gray matter volume than less risk-prone individuals. However, they observed differences between these two groups in the integrity of the white matter in frontal regions. Sakai et al. [17] found that older people with lower executive function had a lower volume in the supplementary motor area (SMA) and, more importantly, were prone to risky driving. Dedovic et al. [18] found that men who had driven under the influence of alcohol (without engaging in other dangerous drinking patterns) showed a reduced cortical thickness of the posterior cingulate cortex (PCC) compared with drivers in the control group. Finally, Aydogan et al. [19] observed that drivers who reported driving faster than the allowable speed limit had lower GMV in the ventromedial and dorsolateral prefrontal cortices, amygdala, and striatum. The evidence gathered to date shows the need to study further the neuroanatomical basis of risk-taking behavior in driving.

Sensitivity to reward (SR) and punishment (SP) reflect individual differences in the behavioral activation system (BAS) and the behavioral inhibition system (BIS), which control the approach and inhibitory responses to appetitive or aversive stimuli [20]. Risky behavior has been linked to greater sensitivity to rewards and less sensitivity to punishment [21]. [22]) found that drivers with high sensitivity to rewards and minor sensitivity to punishment behaved in a riskier way while driving and in health-related behaviors. However, other studies appear to indicate that sensitivity to punishment has little influence on risky driving and that sensitivity to rewards is a distal predictor of this behavior [5, 23, 24]. Therefore, the relationship between sensitivity to reward and punishment and risky driving behavior is still unclear.

Furthermore, the relationships between SR and SP and brain volume in risky driving contexts have not yet been studied, although some studies have explored the association between brain volume and personality traits such as SP and SR or impulsivity. Regarding SR, positive and negative correlations have been found with the volume of the striatum ([25–28]) and negative correlations with the volumes of the lateral and medial prefrontal and superior temporal cortices [25, 27, 29]. On the other hand, SP has been positively correlated with volumes of the amygdala and hippocampal formation and negatively with the insula and OFC volumes [25, 30–35]. Thus, the correlations between brain structure and SR and SP could differ depending on the population under study. In this regard, Parvaz et al. [36] found that the P300 (an event-related measure of reward sensitivity) was positively related to the volume of the frontostriatal circuit in healthy participants. However, in people addicted to cocaine, no relationship was observed between P300 and gray matter volume. Therefore, it is critical to determine whether the relationships between reward and punishment sensitivity and brain gray matter volumes vary depending on whether or not people exhibit risky driving behavior.

Another related and essential personality factor implicated in risk behavior is impulsivity. This personality trait is a multidimensional construct that includes the tendency to choose risky options, the inability to assess the risk associated with a decision, or the preference for immediate reinforcement [37, 38]. The preference for immediate reward in delayed discounting tasks (DDT) has been positively related to risk behavior, such as financial [39] or risky sexual behaviors [40, 41]. In stark contrast, other studies have not observed significant relationships between discounting rate and risk behavior [42, 43]. Regarding risky driving behavior, some studies have found a positive relationship between the value placed on immediate rewards and self-reported risky driving [44, 45] or errors while driving in a simulator [46]. It has also been observed that drivers who use a mobile phone while driving have a higher discounting rate than those who do not [47] although this finding was not replicated in subsequent studies [48]. Furthermore, in a recent study, Qu et al. [49] have observed no relationship between the preference for immediate reinforcement and risky driving behavior. However, these authors demonstrated that a higher discounting rate for large rewards significantly predicted safer driving behaviors. Therefore, the type of relationship between risky driving and a preference for immediate reinforcement seems questionable.

Regarding the brain correlates of cognitive impulsivity, the neural networks involved in valuation (striatum, OFC, medial prefrontal, lateral parietal, and posterior cingulate cortices), conflict monitoring and cognitive control (ACC and LPFC), and prospection (hippocampus and amygdala) have been assumed to underlie the process of delay discounting [50, 51]. Some relationships between the preference for immediate reinforcement and gray matter volumes of various brain areas have been found at the neuroanatomical level. For instance, the positive and negative correlations have been observed between the gray matter volume and the discounting rate in medial prefrontal regions, superior frontal gyrus, OFC, striatum, and ACC ([52–61]). The preference for immediate reinforcement has also been negatively associated with volumes of the lingual gyrus, LPFC, entorhinal cortex, and medial temporal gyrus [62, 63]. Likewise, the positive relationships have been observed between volumes of the parahippocampal gyrus, PCC, insula, and lateral occipital cortex and the discounting rate [61, 64, 65]. Finally, regarding the total gray matter volume, Owens et al. [63] have observed that a higher discounting rate is significantly associated with a lower total cortical, but not subcortical, gray matter. Despite previous evidence, the associations between gray matter volume and delay discounting seem inconclusive and vary depending on the population under study. In this regard, Wang et al. [66] found that while impulsivity was negatively related to the volumes of frontal and limbic areas in healthy people, no such relationship was found in obese individuals.

To the best of our knowledge, no research has yet been done to examine the neuroanatomical correlates of delay discounting in drivers. Therefore, it is necessary to carry out an in-depth study of the associations between preference for immediate reinforcement and cerebral gray matter volume, which could be very helpful for determining whether these associations vary depending on the extent to which drivers are risk-prone. Thus, the main objective of this paper was to study the neuroanatomical bases of risky driving behavior and how the level of risk-taking influences the link between impulsivity and sensitivity to reward and punishment and the volume of brain gray matter. We hypothesized that riskier drivers would have a lower volume of brain gray matter than less risky drivers, particularly in areas related to reward and cognitive control processing and valuation. Furthermore, according to previous literature [36, 66], we expect that the relationship between personality traits and brain gray matter volume depends on the level of risky driving.

## 2. Materials and Methods

### 2.1. Participants

The participants in this study were part of a more extensive study aimed at revealing the brain basis of risk behavior in traffic situations. We used structural MRI from 144 participants (50 women, 32.06 years old, range = [18, 68]). None of the participants reported a history of head injury nor a history of neurological disorders. All participants signed an informed consent form, were informed of their rights, and were treated according to the Helsinki Declaration [67]. All participants were paid for their participation in the study. The Ethics Committee of Human Research of the University of Granada approved this research (204/CEIH/2016). The participants were then organized into three groups, according to their risky driving behavior in real life.

### 2.2. Risk Classification

Each participant was asked to indicate whether and how many points they had lost in the Spanish fine system due to traffic rule violations, whether they have attended a rehabilitation course to recover these points, how many fines they had received for violating traffic rules, and if they usually exceed the speed limit by 20% or higher when driving. All these variables are binary and of different importance, which precludes their use as numerical variables or continuous variables. The non-risk (NR) group was composed of 28 participants who had received up to two fines but had not lost points, had not attended a rehabilitation course, and did not exceed the speed limit by 20% when driving. The medium-risk (MR) group was composed of 53 participants who had retained all their points but had received more than two fines and usually exceed the speed limit by more than 20% when driving. Finally, the High-Risk (HR) group was composed of 63 participants who had lost more than one point from their driver's license due to severe violations of traffic rules.

### 2.3. Instruments

#### 2.3.1. Sensitivity to Punishment and Sensitivity to Reward Questionnaire

The sensitivity to punishment and sensitivity to reward questionnaire (SPSRQ-20; [68]) consists of 20 dichotomic items (Yes/No) divided into two subscales: the sensitivity to reward (SR) and sensitivity to punishment (SP). The SR measures the BAS, and the SP measures the BIS [69].

#### 2.3.2. Monetary Choice Questionnaire

The Monetary-Choice Questionnaire (MCQ; [70]) evaluates individual preferences between smaller, immediate rewards (SIRs) and more significant, delayed rewards (LDRs) that vary in their value and time to be delivered. Participants are presented with a fixed set of 27 choices between SIRs and LDRs. For example, on the first trial, the participants were asked, “Would you prefer 54 euros today, or 55 euros in 117 days?” The trial order was arranged so that it did not correlate with the immediate or delayed reward amounts, their ratio, their difference, the delay to reward, or the discounting rate corresponding to indifference between the two rewards [71]. The preference for immediate rewards is calculated by counting the number of choices of SIRs.

### 2.4. Procedure

The participants came to the research center and, as a part of a broader project, signed the informed consent form, completed the questionnaires, and underwent the MRI scan. The order of the questionnaires and MRI scanning were arranged according to the availability of MRI and the participants' schedules.

### 2.5. MRI and Data Analysis

The MRI scans were conducted with a Siemens 3T Trio system equipped with a 32-channel head coil at the Mind, Brain, and Behavior Research Center of the University of Granada. The participants were instructed not to move during the scan. Head restraint and foam padding around the head were used to limit head motion. A T1-weighted MPRAGE scan was obtained with a TR (repetition time) of 1900 ms, TE (echo time) of 2.52 ms, and a flip angle of 9°. For each volume, 176 slices of 1 mm thickness were obtained, which provide whole-brain coverage (voxel size =1 × 1 × 1 mm; FOV =256 mm; 256 × 256 data acquisition matrix).

The MRI scans were submitted to CAT12 toolbox (http://www.neuro.uni-jena.de/cat/) to obtain brain volumes, running under the umbrella of SPM12 (https://www.fil.ion.ucl.ac.uk/spm/software/spm12/), using default parameters. In essence, CAT12 corrects for bias inhomogeneity, segmented into gray matter, white matter, and cerebrospinal fluid using the AMAP approach, and the images were spatially normalized using the diffeomorphic anatomical registration through the exponentiated lie algebra (DARTEL) algorithm. Volumes were then normalized to the MNI neurological space and multiplied by the Jacobian determinant to preserve volume. Gray matter volumes were then smoothed using an 8 mm FWHM Gaussian kernel. This volumes were submitted to a voxel-wise analysis, as described below. After that, the neuromorphometric anatomical areas were extracted to perform partial correlation analysis (see below for further details).

1SPM 12 was used to perform the voxel-wise statistical analyses. The general linear model was used, in which a single factor (three levels) was manipulated between subjects. The comparisons between the three groups were made while controlling for age, gender, education level, and total intracranial volume (TIV) (results are also provided controlling only for age, gender, and educational level, for sensitivity analysis and comparative purposes). FDR corrected the significance threshold to a cluster *q* < 0.05; we used an extended cluster size of 240 voxels based on simulations done with the Rest-AlphaSim (FWHM =8, mm =4, voxel threshold =0.001), 1000 iterations, to further control for the multiple comparison problem. The automated anatomic atlas (AAL) was used to label the significant clusters of interest.

Our second analysis was aimed at uncovering the relationships between SPSRQ and MCQ scores and the brain, using a partial correlation approach. For this approach, we used the anatomic parcellation provided by the computational anatomy toolbox (CAT12). This software provides a volumetric information according to the neuromorphometric atlas. We obtained the volumes of 116 structures (only regions with gray matter were retained, so 26 of the 142 regions provided by the neuromorphometric atlas were excluded), which were then correlated using the partial correlation coefficients with the SPSRQ and the MCQ variables. This analysis also controlled for age, gender, education level, and TIV (data are also provided controlling only for age, gender, and education level, for comparative purpose). The differences between correlation coefficients were then obtained for the comparisons between non-risk versus medium- and high-risk and medium- versus high-risk groups. It is important to note that the size of the correlation coefficient is dependent on the sample size used to compute it. In line with a recent proposal regarding the significance threshold [72, 73], we adopted a *p* value < 0.005 to test for the statistical significance of these 348 differences.

## 3. Results

Table 1 displays the means and standard deviations for age, education level, TIV, total gray and white matter volumes, the number of women in each group, punishment and reward sensitivity, and the preference for an immediate reward. There were differences in age between group MR and HR (*p* < 0.05) and in the number of women (*p* < 0.05). No other differences were observed. No differences in sensitivity to punishment, sensitivity to reward, or preference for immediate reward were observed between groups (min *p* = 0.11).

No differences in TIV were observed between the three groups (*p* > 0.10). However, differences in total gray matter volume were observed between the NR and HR groups (*p* < 0.01), indicating larger volumes in the NR than the HR group (Table 1). This indicates the general tendency for risky individuals to have a lower total gray matter volume. No differences in white matter volumes were observed between the three groups (all *p* > 0.22).

Table 2 displays the peak *t*-scores for the significant differences, corrected for multiple comparisons. The differences were observed in the left superior parietal cortex for the contrast NR > MR. The differences were also observed in the right parahippocampal gyrus, right cerebellum 6, and left caudate, volumes for the contrast MR > HR. The differences in volumes of the vermis, right middle frontal cortex, and left superior parietal cortex were observed for the contrast NR > HR. Note, however, that a larger set of differences were found significant when no TIV controlling was used.

We then used the neuromorphometric atlas to uncover the relationships between scores on the SPSRQ and the MCQ questionnaires and brain parcels (Table 3, Figure 1). We observed that for the NR-MR contrast, the differences between correlations were significant for punishment sensitivity in the right medial precentral cortex, left superior medial frontal cortex, and right posterior insula, while for the immediate reward, the differences were observed in bilateral nucleus accumbens (nAcc), right amygdala, right lingual, right PCC, and left inferior OFC. For the NR-HR contrast, the differences were observed for the reward sensitivity in the left frontal operculum, left medial postcentral cortex, and left superior temporal cortex (STC), while for the immediate reward, the differences were observed in left nAcc and left inferior OFC. Finally, for the MR-HR contrast, the differences were observed for punishment sensitivity in the bilateral medial precentral, reward sensitivity in the left occipital fusiform, and immediate reward in the left occipital pole and left PCC. Note that when no TIV control was applied, fewer brain areas remained significant.

## 4. Discussion

In the present research, we studied the anatomical bases of risky driving behavior and its relationships with reward and punishment sensitivity and the tendency to delay rewards. The main findings are that total gray matter volume varies as a function of risk proneness, with lower brain gray volumes related to higher risk tendencies. This finding applies to both total gray matter volumes and volumes of the frontotemporal, parietal, limbic, and cerebellar cortices (the total number of areas varies according to TIV control). The relationships between reward and punishment sensitivity and the ability to delay rewards and gray matter volumes differ as a function of risk tendency. High-risk individuals showed, in general, lower absolute correlations with gray matter volumes than the less risk-prone individuals. We have also shown that the level of risk is the main factor modulating the relationship between personality traits and brain gray matter volume. When the TIV control was applied, the relationship between preference for immediate reward and gray matter volume was observed to differ between the NR and MR groups in the nAcc, amygdala, lingual gyrus, inferior OFC and PCC, between the NR and HR groups in the left hemisphere structures (nAcc, inferior OFC), and between the MR and HR group in the occipital pole and posterior cingulate cortex. The relationships between sensitivity to punishment and brain gray matter volume also differed between the NR and MR groups in the right medial precentral cortex, left superior medial frontal cortex and right posterior insula, and between the MR and HR groups in the bilateral medial precentral cortex. Finally, the partial correlation between reward sensitivity and gray matter volume differed significantly between groups NR and HR in the left frontal operculum, left medial postcentral and left STC, and between groups MR and HR in the left occipital fusiform cortex. When no TIV control was applied, fewer brain areas remained significant.

It is important to note that the use of two different control strategies, including or not the TIV as a covariate, has been done for comparative and sensitivity analysis purposes. The robustness of the data is confirmed by the fact that the control, or not, of the TIV does not modify the type of structure in which differences are found, but rather increases or decreases the significance of these differences. Regarding the study of the anatomical bases of risky driving, both analyses result in differences in GMV between the groups in the same structures. When controlling for TIV, some differences are no longer significant, but no new structures appear, nor is the directionality of the differences reversed. Previous studies confirm our results by finding that the different TIV adjustment methods provide different results and these do not only eliminate the GMV differences between groups, but rather make them smaller and in a fewer structures [74–76]. Something similar occurs when using the partial correlation coefficient to study the relationships between GMV and personality traits as a function of risk level. When controlling for TIV, significant relationships appear that were not previously significant and those that were already present when TIV was not taken into account are maintained. Previous studies have also found differences in the statistical power of the relationships between personality traits and GMV depending on the control variables used [74, 77, 78]. The point that when not controlling for TIV our results show a reduction in the number of structures that are related to personality traits may be due to the fact that these relationships appear but cannot be observed because they are masked by a TIV that is not being taken into account.

### 4.1. Risk-Proneness in Driving Depends on Differences in GMV

Our results demonstrate that risky drivers have a lower total gray matter volume than non-risky drivers. This negative relationship between brain total gray matter and risky behavior has also been observed in other measures of risky behavior, such as early use of addictive substances [79]. Regarding the brain areas, before controlling the TIV we have observed that the riskiest drivers have lower gray matter volume in the left superior frontal cortex, medial frontal cortex, triangular inferior frontal cortex, medial and inferior orbital frontal cortex, superior temporal cortex, temporal pole, superior parietal cortex, cerebellum, fusiform gyrus, insula, parahippocampus, caudate and putamen. The superior parietal and medial frontal cortices, cerebellum, parahippocampus, and caudate remained significant after controlling the TIV.

Some of these regions, such as the OFC, the parahippocampus, the caudate, or the putamen, are part of the brain's socioemotional or reward system [50, 80–87]. This system is involved in the sensitivity, detection, and processing of incentive signals; the prospection and representation of reward expectations based on previous experience; and in the search, evaluation, and approach to reinforcers [11, 82–84, 87–89]. Thus, our results suggest an alteration in the detection, processing, and valuation of rewards in the riskiest drivers, which may involve maladaptive decision-making in traffic situations.

On the other hand, other regions in which we observe lower gray matter volume in risky drivers, such as the superior, medial, and inferior frontal cortex, the superior and medial temporal cortex, the fusiform gyrus, the cerebellum, and the superior parietal cortex, are part of the cognitive control network [85, 86, 90–96]. This network is responsible for controlling the general implementation of tasks, particularly during the decision-making phase in probabilistic or intertemporal choice tasks [90, 92]. More specifically, this network is involved in the identification of stimuli relevant for the task, inhibitory and attentional control, working memory, conflict and error monitoring, and self-regulation of behavior [85, 86, 90–94, 96, 97]. These executive functions related to cognitive control have been associated with better execution of driving and less risky behavior while driving [98–105]. Thus, consistent with the previous literature, our results indicate an alteration in cognitive control processes in risky drivers, resulting in risky driving decisions.

The reduced volume of brain structures in risky drivers could alter the reward and cognitive control brain networks. These networks act as a dual neurobiological system that works interactively to modulate the decision-making process [106]. On the one hand, the socioemotional system processes the reinforcers and biases decision-making based on assessing and predicting possible rewards and punishments. On the other hand, the cognitive control system is involved in the selection of actions, conflict monitoring, impulse inhibition, and regulation of the influence of the reward system on the decision-making process [36, 50, 52, 84, 87, 107–110]. Gray matter volume alterations in these areas have been described in executive functioning alterations [111] and manifestations of risk behavior in both self-reported and laboratory tasks [106, 109, 112–114].

With regard to driving, Beeli et al. [115] observed that transcranial magnetic stimulation of the LPFC, one of the most critical areas in the cognitive control system, caused drivers to behave in a less risky way (as measured by speed, distance from another car, and speed violations) while driving in a simulator. In another study, Chein et al. [107] found that adolescents presented more extensive activation of the brain regions involved in reward and took more risks in a driving game in the presence of peers. Moreover, compared with adults, they showed less activation of the regions related to cognitive control. However, adolescents with greater activation of the control network behaved more safely while driving [116]. On the other hand, Aydogan et al. [19] have found that people who reported higher risk behavior related to alcohol, smoking, sex, or driving had a lower gray matter volume in areas such as the striatum, putamen, ventromedial, and dorsolateral prefrontal cortex, insula, and cerebellum. In another recent study, Yamamoto et al. [117] have evaluated, using realistic driving situations, risky driving at intersections with stop signs in a group of older adults without cognitive impairment. The best predictors for classifying risky and non-risky drivers were age and the gray matter volume of areas related to executive functions, cognitive control, and incentive processing in the frontal and parietal cortices. These studies support our results regarding the negative relationship between risky driving and gray matter volume of the areas involved in the reward and cognitive control circuits.

The reduced volume of brain structures in risky drivers could also be related to different functionality since any alteration of gray matter volumes appears to influence functional neural activity [118]. Aydogan et al. [19] compared their results on brain structure and risk behavior with a meta-analysis of functional magnetic resonance imaging and risk behavior studies (https://neurosynth.org/). These authors observed that many brain structures that were anatomically associated with risk behavior were also functionally related to such behavior. On the other hand, a wide variety of studies have observed differential brain activation when performing various laboratory tasks depending on the individuals' level of risk proneness [9, 88, 119–121]. These results show that people who engage in risky behaviors, such as reckless driving, could use a different distribution of cognitive resources to non-risky people.

Thus, our results suggest that, in risky drivers, there is an alteration at the level of brain structure in the neural circuits involved in reward processing and cognitive control. Furthermore, these alterations could reflect a distinctive brain activation pattern, which could imply that these drivers show maladaptive information processing and dysfunctional decision making [21, 120].

### 4.2. Personality Factors and Risk Driving

Regarding the sensitivity to rewards and punishments, our results are in line with those obtained by Brown et al. [122]. These authors examined the personality characteristics of three different forms of risky driving: driving while impaired (alcohol-related traffic offenses), speed (non-alcohol-related traffic offenses), and mixed (alcohol-related and speed-related traffic offenses). They found no differences in SPSRQ scores between any of the groups and the control group (no traffic offenses), except for the mixed group, which showed greater sensitivity to rewards than the control group. In another study with repeat offenders, Padilla et al. [5] have found that sensitivity to rewards, but not sensitivity to punishment, acted as a distal predictor of recidivism. In reference to other risk behavior measures, Navas et al. [123] found that, although obese people made riskier choices, there were no differences between them and the control group in terms of SPSRQ scores.

Regarding impulsivity, our results are consistent with those obtained by Qu et al. [49], who found no significant relationships between the preference for immediate reinforcements and risky driving behavior. Hlavatá et al. [124] investigated the relationship between impulsivity and impulse control disorder in a group of patients with Parkinson's disease. They found that, although the experimental group differed from the control group in self-reported impulsivity and risk behavior, the groups did not differ in DDT scores. In another study with Parkinson's disease patients, no relationships were observed between performance on various tasks that measure risk behavior (BART; IGT) and DDT [125].

However, many studies have found relationships between personality traits and risk behavior [21, 22, 39, 46]. It seems that the association between risk behavior and certain personality factors, such as sensitivity to rewards and punishments or cognitive impulsivity, may depend on the dimension of risk evaluated and the population under study.

In this vein, it is essential to note that most studies that have found relationships between risky driving and SPSRQ or delay discounting scores evaluate driving risk through self-report measures [22, 44, 45]. We have used a more ecological measure to determine individual risk proneness (points lost from the driver's license, attendance to recovery courses, fines for traffic violations, and driving over the speed limit), which can influence how risky driving relates to the different personality measures.

### 4.3. Risk as a Modulator of the Relationships between Personality Factors and Brain Gray Matter

Our results show that the relationship between sensitivity to reward and punishment and impulsivity and brain gray matter are different for different levels or risky driving. In the absence of risk, these personality factors are positively or negatively related to the volume of brain areas involved in cognitive control and incentive processing. However, for medium and high-risk drivers, the association between gray matter volume and impulsivity and reward or punishment sensitivity disappears or is reversed.

Differences in the association between gray matter volume and personality variables were found in the absence of significant group differences in the SPSRQ and MCQ scores. Therefore, it seems that these significant differences between the correlation coefficients of the groups genuinely indicate how the brain gray matter volume of the areas involved in decision-making-related vary as a function of the risk proneness of the drivers. This could mean that risky drivers process information differently to non-risky drivers. This notion is in line with the results reported by Delgado-Rico et al. [126], who found no differences in a risky decision-making task between obese people and healthy controls. However, during the execution of the task, they observed significant differences between the groups in terms of brain activation in the insula and midbrain.

We observed, after controlling also the TIV, a negative relationship between preference for an immediate reward and cerebral gray matter volumes of the nAcc, amygdala, OFC, PCC, and lingual gyrus, but a positive relationship between this preference and occipital cortex volume in less risky drivers. However, this relationship either disappears or is reversed in the riskiest driver groups. Previous studies have shown that these brain areas are included within the neural networks associated with the delay discounting process. [50, 51]. The nAcc is part of the ventral striatum, which is involved in the sensory processing and valuation of rewards and the anticipation and learning of reinforcement [81, 84, 89, 127]. Rats with lesions in this area were found to make fewer good choices and showed a decrease in gain rates on delay discounting tasks [128]. The OFC integrates the information from the limbic areas to determine the value of rewards and to control the decision-making process [85, 87, 129]. Several studies have linked the gray matter volume of the OFC with cognitive impulsivity or sensitivity to immediate reinforcements ([54, 64]; Li et al., 2019; [65, 130]). The PCC, which is connected to the OFC and is part of the DMN, is also involved in the subjective value of rewards and is responsible for responding to environmental variations that require behavioral change [50, 131–133]. The structure and activation of the PCC have been related to the decision-making process in delay discounting tasks [51, 59, 134, 135]. Furthermore, Dedovic et al. [18] have found a reduced cortical thickness in this area in men who had driven under the influence of alcohol. Regarding the occipital cortex, structure and functional connectivity data have related this area to delay discounting rates [61, 65].

Our results agree with those observed on the neural networks involved in delay-discounting and suggest that the trait-structure association could be altered in risky drivers. Numerous studies have concluded that, in pathological gamblers and patients with other psychiatric disorders, there is an alteration in the processing and decision-making related to the delay discounting process, as reflected in activation patterns and differential brain structure, when compared with healthy controls (for a review, see Noda et al. [136]. More specifically, Hobkirk et al. [137] found that, in cocaine users, the delay discounting rate was not related to resting-state functional connectivity between the reinforcement and attentional salience networks, a correlation that was significant in the control group. On the other hand, Wang et al. [66] observed that impulsivity was negatively related to the gray matter volume of areas responsible for cognitive control and incentive processing in healthy people. However, similar to our results, this relationship disappeared in obese people, and this occurred in the absence of significant differences between groups on the impulsivity measure. In a similar vein, Freinhofer et al. [55] examined the relationship between DDT performance and brain gray matter volume in a group of patients addicted to gambling and a control group. These authors observed a negative correlation between gray matter volume of the medial OFC and the choice of immediate reinforcement in the control group, a relationship that disappeared in the group of patients addicted to gambling. Furthermore, they found no associations between the performance on a risky decision-making task and discounting delay scores in the whole sample. Therefore, our results support the idea that there is an alteration in the relationship between delay discounting and brain gray matter in various manifestations of risky behavior, such as risky driving.

Regarding the relationship between reward sensitivity and brain gray matter, we observed, after controlling also the TIV, that the former is positively related to the volume of the STC, occipital fusiform gyrus, and medial postcentral gyrus, but negatively related to the left frontal operculum, in less risky drivers. However, this relationship was almost non-existent in the riskiest driver groups in all comparisons. Similarly, in less risky drivers, sensitivity to punishment was negatively related to the gray matter volumes of the insula, the superior medial frontal cortex, and the medial precentral gyrus. Again, these relationships were lost or reversed in medium or high-risk level drivers.

The STC is involved in controlling the decision-making process by integrating the results of previous actions, particularly when these entail rewards [138]. The functional connectivity of this area, such as the nAcc, has been specifically related to sensitivity to music reinforcement [139]. Other authors find that the reward sensitivity is negatively related to the gray matter volume of the STC and, therefore, with poorer cognitive control [25]. The pre- and postcentral gyrus and the fusiform gyrus have been related to the behavioral activation and inhibition systems and have been implicated in the responses to reinforcing and aversive stimuli [31, 140–145]. More specifically, Sakai et al. [17] show that, in older people, the volume of the SMA is a good predictor of individual differences in executive functions and these act as a risk factor for traffic accidents. The insula and the superior frontal cortex are part of the cognitive control network necessary for driving [146]. These areas are responsible for the identification of the relevant stimuli, the integration of interoceptive stimuli, the prediction of the error to obtain reinforcement or avoid damage, the inhibition of responses, and the behavioral regulation [93, 94, 109, 110, 147]. Von Siebenthal et al. [35] found that the activation of the insula during the decision phase of a roulette task was negatively related to punishment sensitivity, regardless of the value of the outcome. These authors explain the negative correlation between insula volume and sensitivity to punishment by relating sensitivity to punishment with pessimism and with the certainty of obtaining negative results. Sensitivity to punishment has also been negatively related to the activation of the superior frontal cortex in people with the borderline personality disorder and healthy controls [148].

Our results agree with the previous evidence on the neural networks involved in reward and punishment sensitivity and suggest that the trait-structure association could be altered in risky drivers. Previous studies on other manifestations of risk behavior support this idea. Parvaz et al. [36] found that the P300 potential, used as a measure of sensitivity to reinforcement, was positively related to volumes of prefrontal regions involved in the brain's reward system in healthy controls. However, no such relationship was found in people addicted to cocaine. In another study, Moreno-López et al. [149] observed a negative correlation between the volume of the somatosensory cortex and sensitivity to reinforcement in healthy controls. However, this relationship disappeared for obese participants. Furthermore, they also found no differences between the groups in terms of the SPSRQ scores.

Taken together, our results show that the differences observed in the relationships between sensitivity to reward and punishment and delay of reward and brain gray matter volumes, as a function of risk level, could reflect a structural alteration and a change in the neural mechanism underlying these personality traits [66]. In other words, in risky drivers, it seems that the function of brain regions involved in reward and punishment sensitivity and impulsivity is masked by the specific mechanisms involved in risky behavior, which has been demonstrated in functional connectivity studies [21]. Our results support this idea, since the gray matter volumes of many of these brain regions, such as the striatum, OFC, STC, fusiform gyrus, lingual gyrus, and insula, are lower in riskier drivers.

### 4.4. Conclusions

Our results show that drivers with a high-risk proneness in traffic situations have a lower total gray matter volume. We have also found that risky drivers have lower gray matter volume in the brain structures responsible for cognitive control and incentive processing. On the other hand, we found that it is the level of risk that determines how these areas are related to personality factors such as impulsivity and sensitivity to reward and punishment. This suggests that, in risky drivers, there is an alteration in the brain structure of the areas involved in reward processing, cognitive control, and behavioral modulation, which could indicate dysfunctional decision-making and riskier driving behavior.

## Figures and Tables

**Figure 1:** An illustration of the correlations between the brain parcels (left accumbens, left inferior frontal orbital gyrus, and right posterior insula) and preference for immediate rewards (IR) and sensitivity to punishment (SP) for each risk group.

**Table 1:** Means and standard deviations for age, education level, number of women, total intracranial volume, total gray and white matter volumes, punishment and reward sensitivity, and preference for immediate rewards in each group.

Group	Age	Education	Gender	TIV	GMV	WMV	SP	SR	IR	N
NR	30.8 (14.9)	3.5 (0.5)	*F* = 9	1614.1 (134.7)	741.5 (66.5)	540.4 (62.4)	2.9 (2.3)	4.4 (2.2)	15.0 (5.0)	28
MR	25.6 (10.7)	3.6 (0.5)	*F* = 30	1541.7 (139.6)	722.4 (73.3)	511.0 (56.1)	3.9 (2.9)	4.4 (2.6)	14.2 (4.5)	53
HR	38.1 (12.4)	3.3 (0.8)	*F* = 11	1565.6 (116.8)	692.1 (60.3)	532.2 (52.8)	3.4 (2.7)	3.8 (2.8)	14.9 (5.5)	63

Note NR: non-risk; MR: medium-risk; HR: high-risk; TIV: total intracranial volume; GMV: gray matter volume, WMV: white matter volume; SP: sensitivity to punishment, SR: sensitivity to reward; IR: immediate reward.

**Table 2:** Between-group comparisons in brain gray matter volume, adjusted for age, sex, and cultural level (left) and also by total intracranial volume (right).

Label	Controlled by age, sex, education						And TIV	
	Size	*t*-peak	*X*	*Y*	*Z*	pFDR	Size	pFDR
NR > MR								
Parietal_Sup_L	1138	4.48	-33	-41	63	0.001	793	0.001
MR > HR								
ParaHippocampal_R	2355	4.72	47	5	-47	0.001	1250	0.001
Cerebellum_6_R	926	4.09	26	-48	-27	0.001	318	0.03
Caudate_L	660	4.01	-14	27	0	0.001	245	0.05
Putamen_R	430	3.9	35	2	0	0.01		
SupraMarginal_R	337	3.64	59	-30	35	0.023		
NR > HR								
Cerebellum_6_R	2014	4.17	35	-71	-30	0.001		
Cerebellum_9_L	412	3.72	15	-57	-56	0.005		
Cerebellum_Crus2_l	819	4.15	-45	-62	-26	0.001		
Vermis_1_2	1808	4.63	-15	-44	-23	0.001	527	0.004
Frontal_Inf_Orb_L	388	4.03	-53	42	-5	0.006		
Frontal_Inf_Tri_R	502	4.35	41	17	17	0.002		
Frontal_Med_Orb_L	364	3.49	15	5	-17	0.007		
Frontal_Mid_L	1741	4.53	-50	8	39	0.001		
Frontal_Mid_R	3940	4.97	27	29	41	0.001	335	0.014
Frontal_Sup_Medial_L	495	4.13	-5	56	32	0.002		
Fusiform_R	512	3.82	45	0	-51	0.002		
Heschl_R	368	4.17	63	-11	9	0.007		
Insula_R	1170	4.74	36	-5	-2	0.001		
Lingual_L	1087	4.71	-24	-90	-6	0.001		
Parietal_Sup_L	3092	4.69	-35	-39	53	0.001	435	0.006
Temporal_Sup_R	1087	4.64	59	-27	30	0.001		
Temporal_Sup_L	461	3.95	-41	14	-14	0.003		
Temporal_Pole_Mid_R	2375	4.13	45	21	-5	0.001		

Note:NR: non-risk; MR: medium-risk; HR: high-risk.

**Table 3:** Between-groups contrast of the correlations between SPSRQ and MCQ scores and gray matter volume, after controlling for age, sex, and cultural level (left) and also by total intracranial volume (right).

Variable	Controlling for age, sex, and cultural level				And for TIV		
	Label	*r*1	*r*2	*z*	*r*1	*r*2	*z*
NR-MR							
IR	L accumbens	-0.54∗	0.18	-3.24	-0.57∗	0.26∗	-3.73
IR	R accumbens				-0.48∗	0.14	-2.73
IR	R amygdala				-0.25	0.39∗	-2.69
IR	R lingual				-0.34∗	0.40∗	-3.18
IR	L inferior frontal orbital	-0.63∗	-0.04	-2.86	-0.68∗	0.00	-3.40
IR	R posterior cingulate				-0.31∗	0.36∗	-2.88
SP	R medial precentral				0.32∗	-0.34∗	2.80
SP	L superior medial frontal				-0.59∗	0.02	-2.85
SP	R posterior insula	-0.5∗	0.14	-2.83	-0.45∗	0.26∗	-3.09
NR-HR							
IR	L accumbens				-0.57∗	0.04	-2.89
IR	L inferior frontal orbital	-0.63∗	-0.11	-2.65	-0.68∗	0.01	-3.51
SR	L frontal operculum				-0.42∗	0.17	-2.61
SR	L medial postcentral	0.43∗	-0.2∗	2.8	0.43∗	-0.22∗	2.90
SR	L superior temporal				0.50∗	-0.08	2.63
MR-HR							
IR	L occipital pole	0.23∗	-0.3∗	2.86	0.35∗	-0.18	2.85
IR	L posterior cingulate	0.25∗	-0.27∗	2.76	0.42∗	-0.10	2.88
SP	L medial precentral	-0.38∗	0.27∗	-3.53	-0.36∗	0.30∗	-3.60
SP	R medial precentral				-0.34∗	0.15	-2.62
SR	L occipital fusiform	0.37∗	-0.13	2.71	0.38∗	-0.14	2.80

Note: NR: no-risk; MR: medium-risk; HR: high-risk; *r*1 is the relationship between the first term of the comparison and the volume of gray matter, *r*2 is the relationship between the second term of the comparison and gray matter; SR: sensitivity to reward, SP: sensitivity to punishment, IR: immediate reward score. ∗These correlations were significant at an uncorrected *p* < 0.05. The differences between correlations were significant at *p* < 0.005.

## Data Availability

The raw data supporting the conclusions of this article are not able to be made openly available because the participants did not give consent to do so.
